# COVID-19 Vaccine, TRIPS, and Global Health Diplomacy: India's Role at the WTO Platform

**DOI:** 10.1155/2021/6658070

**Published:** 2021-08-26

**Authors:** Vijay Kumar Chattu, Bawa Singh, Jaspal Kaur, Mihajlo Jakovljevic

**Affiliations:** ^1^Division of Occupational Medicine, Department of Medicine, Faculty of Medicine, University of Toronto, Toronto, ON, Canada M5G 2C4; ^2^Department of Public Health, Saveetha Medical College, Saveetha Institute of Medical and Technical Sciences, Saveetha University, 600077, Chennai, India; ^3^Institute of International Relations, The University of the West Indies, St. Augustine, Trinidad and Tobago; ^4^Department of South and Central Asian Studies, School of International Studies, Central University of Punjab, PIN-151401, Bathinda, India; ^5^Department of law, Guru Nanak Dev University, Regional Campus, Jalandhar, Punjab 144007, India; ^6^Department of Global Health Economics and Policy, Faculty of Medical Sciences, University of Kragujevac, Kragujevac 34000, Serbia; ^7^Institute of Comparative Economics, Hosei University, Tokyo 194-0298, Japan; ^8^Department of Public Health and Healthcare named after N.A. Semashko I.M. Sechenov First Moscow State Medical University (Sechenov University), Moscow, Russia

## Abstract

In light of the devastation caused by COVID-19, the Agreement on Trade-Related Aspects of Intellectual Property Rights (TRIPS) and vaccine research and development (R&D) have been occupying a prominent position in the field of global health diplomacy (GHD). Most countries, international organizations, and charitable organizations have been engaged in the R&D of COVID-19 vaccines to ensure timely affordability and accessibility to all countries. Concomitantly, the World Trade Organization (WTO) provides some provisions and enforcements regarding copyrights, patents, trademarks, geographical indications, and industrial designs. Given these safeguards, it is considered that intellectual property rights (IPRs) have become major barriers to the affordability and accessibility of vaccines/medicines/technology, particularly to the developing/least developed countries. Realizing the gravity of the pandemic impact, as well as its huge population and size, India has elevated this issue in its global health diplomacy by submitting a joint proposal with South Africa to the World Trade Organization (WTO) for a temporary waiver of IPRs to ensure timely affordability and accessibility of COVID-19 medical products to all countries. However, the issue of the temporary waive off had become a geopolitical issue. Countries that used to claim per se as strong advocates of human rights, egalitarianism, and healthy democracy have opposed this proposal. In this contrasting milieu, this paper is aimed at examining how the TRIPS has become a barrier for developing countries' development and distribution of vaccines/technology; secondly, how India strategizes its role in the WTO in pursuant of its global health diplomacy? We conclude that the IPRs regime should not become a barrier to the accessibility/affordability of essential drugs and vaccines. To ensure access, India needs to get more engaged in GHD with all the involved global stakeholders to get strong support for their joint proposal. The developed countries that rejected/resisted the proposal can rethink their full support.

## 1. Introduction

In the context of COVID-19, the Agreement on Trade-Related Aspects of Intellectual Property Rights (TRIPS) has been identified as one of the most significant barriers to vaccine and medicine affordability, particularly for developing and least developed countries. TRIPS is a hard law instrument that is enforceable and binding; it mandates patent protection for pharmaceutical products for up to 20 years, and any violations result in trade sanctions [1]. Apart from the lack of pharmaceutical research and development (R&D), patents on pharmaceutical products and processes and poverty used to become double whammies for third world countries. Given the monopolies over vaccine production, marketing and fixing the higher prices maximize profits by the multinational pharmaceutical and drug companies/developed countries. Global health diplomacy is an integral part of Indian foreign policy. Recognizing the urgency of the situation, India and South Africa have jointly submitted a draught request to the World Trade Organization (WTO) for a temporary waiver of intellectual property (IP) rights to make COVID-19 medications affordable and accessible to all. [2]. In this scenario, the main focus of this paper is to examine how the pharmaceutical TRIPS have become a barrier to the development and distribution of vaccines/technology to the poor countries. The paper also argues why the developed countries (advocates of health, democracy, egalitarianism, and protection of human rights) are refusing to support the temporary IP waiver proposal for the humanitarian cause. Even though international trade cooperation has suffered from geopolitical shifts and competition in the midst of the pandemic crisis, governments can align their trade and health policies to serve the global community by engaging in GHD [3].

Because of this COVID-19 pandemic and the consequent lack of vaccines/medicines, many developed countries are actively engaged in vaccine R&D. According to recent findings from a country pandemic risk exposure measurement model, the national risk management strategies in Italy and Spain have anticipated these needs [4]. On the contrary, public criticism in many developing nations has grown exponentially, as issues about the legitimacy of patents on life-saving vaccines have been raised. This has contributed to the call for modifications or amendments to the TRIPS, which many claims are too strongly favoring private and commercial rights and interest, and against public interests. However, developing countries such as India and South Africa, which are seen as the emerging leaders of third world countries, are concerned that TRIPS may prevent the patients from these countries' from accessing essential COVID-19 vaccines/medicines/technologies. Given this context, we conducted a review to examine how TRIPS has become a barrier to the development and distribution of vaccines/and technology in developing countries. Second, we looked at how India strategizes its involvement in the WTO through its global health diplomacy.

## 2. Methodology

A literature search was done in all the major databases, namely, PubMed, Web of Science, Scopus, and Google search engine for the terms “COVID-19” OR “COVID-19 Vaccine” OR “Trade-Related Aspects of Intellectual Property Rights (TRIPS)” OR “World Trade Organization” OR “Global Health Diplomacy” AND “India.” All relevant titles were screened, and essential information was extracted in preparation for this review. A total of 40 full-text articles and eight other reports were reviewed, and the findings are discussed in three main sections, namely, (1) COVID-19 medical products and TRIPS, (2) COVID-19 Vaccine and TRIPS, and (3) Global Health Diplomacy: India's Role at the WTO Platform.

## 3. Results

### 3.1. COVID-19 Medical Products and TRIPS

The economic and social disruptions caused by the COVID-19 pandemic are devastating. Millions of people are at the risk of falling into extreme poverty. Globally, there have been 115,653,459 cases, including 2,571,823 deaths reported to WHO as of March 6, 2021 [5]. It had become a critical challenge for the developing and least developed countries where healthcare systems are not adequate to care for the affected people. With its great toll of lives and strain on the healthcare systems, COVID-19 has been a great challenge for such countries and even the developed countries. On December 2, 2020, WHO has published its official release of “Draft Landscape of COVID-19 Candidate vaccines 2020,” which contained a total of 51 Candidate Vaccines in Clinical Evaluation with more additions coming in [6]. Treatments available for patients suffering from an active clinical form of the disease also remain scattered and without firm consensus on efficiency ranging from old antimalarial drug chloroquine [7] over convalescent plasma [8] up to novel targeted monoclonal antibodies [9]. Secondly, it had left indelible imprints on unemployment, poverty, hunger, undernourishment, etc. Thirdly, whatever the efforts are being made for vaccines R&D [10] that would likely remain beyond common people's reach, given the high prices of the same due to TRIPS. A number of studies have already proven that the most developed non-OECD South Asian countries confront significant impediments to the financial affordability of pharmaceuticals for the general public, even in the richest coastal and metropolitan districts of their major cities [11]. Now, how TRIPS is one of the major concerns for the availability of the medicines is the moot question in this context?

The intellectual property rights (IPRs) started taking place during the late 19^th^ century, formally concretized in 1995. The IPRs are meant for protecting the creators/agencies' exclusive rights over the creation/s for a certain period. While the agreement establishes minimum standards for intellectual property right (IPRs) protection in the form of patents, trademarks, geographical indications, industrial designs, and the enforcement of those rights in all WTO member countries, it is primarily concerned with reducing distortions and impediments to international trade.

The TRIPS has been conceived very beneficial for society, particularly given the imposition of temporary monopolies and other limitations resulting from private IPRs [12, 13]. By putting legal protections in place and tackling piracy and counterfeiting through the IPs, the creation of new knowledge, innovation, and creativity is being encouraged. Therefore, the costs associated with the R&D can be retrieved, and remuneration would be earned. Matthews [14] argues that the IP regime not only stimulates domestic innovation but also promotes knowledge diffusion, technology transfer and licencing, and Foreign Direct Investment (FDI) to developing and least developed countries, thereby promoting trade and economic development in those countries. On the contrary, Sell and Prakash [1] have argued that the TRIPS has also been subjected to severe criticism since their inception. Recently, on October 16, 2020, during the WTO TRIPS Council meeting, nine WTO members, including the European Union, did not support the proposal though 100 countries showed support for the proposal. Though Canada became the first country worldwide to reform its domestic law to enhance developing countries' access to patented medicines [15], it did not support the IP waiver proposed by India and South Africa recently in October 2020. It was proposed that Canada should assist developing countries in their calls for greater access to existing pharmaceuticals and technologies, as well as access to new treatments and equipment. Furthermore, it is an excellent time for global solidarity, and Canada should take advantage of this chance to reassess its position on IP acquisition in relation to other domestic and international policy levers [16].

### 3.2. COVID-19 Vaccines and TRIPS

Since the introduction of research and development in the biological sciences, vaccines have been given a vital place and role in saving millions of lives each year. Vaccines are used to prepare the body's natural immune system to combat viruses and bacteria. On December 2, 2020, WHO published its official release of “Draft landscape of COVID-19 candidate vaccines 2020,” which contains a list of 51 candidate vaccines in clinical evaluation [6]. Yet, we mentioned ongoing efforts to foster early marketing approvals by shortening phase III development duration, with the first global official launch in Russia [17] for emergency use authorization. However, it has not received fully marketing approval in Russia. Similar accelerated development pathways currently occur in the US, China, India, Germany, UK, and possibly Israel [18]. Against this backdrop, the COVID-19 vaccine R&D program has been ongoing at an unprecedented pace to make a preventable disease vaccine [19]. Even assuming this ends up with several agents of acceptable efficiency–toxicity profile, it remains an open-ended question of public acceptance of massive vaccination. Public opposition to such an epidemiological strategy to achieve herd immunity is notable globally, with a huge population of Pakistan being a convenient example [20].

Many scholars such as Thanh et al. [21] and Fau et al. [22] argued that soon after coronavirus detection in December 2019, the genetic sequencing of COVID-19 was published on January 11, 2020 which has necessitated an urgent international reciprocation to develop a preventive vaccine immediately. Schmidt [23] has reported in one of his opinions that about 80 companies, and institutes in 19 countries have been engaged in COVID-19 vaccine R&D. According to Thanh et al. in their report in the Coalition for Epidemic Preparedness Innovations (CEPI), in terms of R&D of COVID-19 vaccine from a geographical standpoint, North America covers 40%; Europe covers approximately 26%; and South America, Africa, Asia, and Australia collectively cover only 30%. These figures indicate that the developed countries monopolize the R&D of the vaccine.

International organizations have taken the lead in this direction and formed international alliances to expedite the R&D of vaccines. International organizations such as the World Bank, WHO, along with the Bill and Melinda Gates Foundation and other International NGOs, have raised a fund of US$ 8.1 billion and introduced the WHO COVAX plan for the fair and equitable distribution of an eventually licensed vaccine. CEPI has also created another fund of US$2 billion from the global partner for the fast-tracked research and clinical testing. Several countries like Belgium, Canada, Germany, Norway, the Netherlands, Switzerland, the UK, and charitable organizations like The Bill and Melinda Gates had contributed about US$ 915 and US$250 million, respectively, in support of CEPI research and public education support for COVID-19 vaccines [24]. In these times, where vaccine nationalism is on the drive due to the scarcity of vaccines, initially, the COVAX initiative is an instrument for a fairer global distribution [25]. Concomitantly, the Global Research Collaboration for Infectious Disease Preparedness (GLoPID-R) and the International Severe Acute Respiratory and Emerging Infection Consortium have been working toward COVID-19 research and eventual vaccine distribution. A virtual summit was organized with private and government representatives of 52 countries, including 35 heads of state from G7 and G20 nations, who supported the Global Alliance for Vaccines and Immunization (GAVI). For example, the European Commission had invested about €80 million in CureVac. Here, we must emphasize a crucial role in global health funding by a set of huge non-OECD actors nicknamed Emerging Markets. Notably, the five nations have been known under the acronym BRICS (Brazil, Russia, India, China, South Africa) or Emerging Markets Seven (EM7-Brazil, Russia, India, China, Mexico, Indonesia, Turkey) [26]. Real GDP growth rates among the EM7 remained substantially higher than G7 during the entire decade of the last global macroeconomic crisis, 2007-2016. Worldwide economic growth accelerating again in 2017 had roughly half of this growth being attributable to the EM7 and only one quarter to the G7 nations. Thus, the health sector's investment and their huge impact on the demand and supply of medical goods and services during the COVID-19 pandemic period shall play an inevitably colossal role. Furthermore, these long-term health expenditure trends are likely to become even more prominent as we approach the mid-2020s as per some prominent forecasts [27].

Some countries have been working in the direction of developing COVID-19 vaccines. The Canadian government pooled about CA$ 275 million for 96 vaccine research projects at Canadian companies and universities, along with a commitment for CA$ 850 million to the WHO for COVID-19 vaccines and preparedness [28]. The Chinese government has been providing low-rate loans to vaccine companies and research institutes. It had also pledged on May 18 to provide about US$ 2 billion to the WHO for the latter's COVID-19 vaccine plans, as well as a US$ 1 billion loan to Latin America and the Caribbean countries to make its vaccine accessible [29]. France had committed a US$ 4.9 million investment in COVID-19 vaccine research undertaken by the CEPI. Germany committed to investing about €300 million investment in CureVac. Several countries like Belgium, Canada, Germany, Norway, the Netherlands, Switzerland, and the UK had contributed about US$ 915 for the COVID-19 vaccines. The other vaccines rolled out with more support from the EU, US, and the UK that are from the Pfizer/BioNTech, AstraZeneca, Moderna, and Johnson & Johnson in early 2021.

The US's federal agencies like Biomedical Advanced Research and Development Authority (BARDA) had announced that about US$ 1 billion would be invested in vaccines. An additional amount of US$ 4 billion would be spent on vaccine development with companies like Sanofi Pasteur and Regeneron. The “Operation Warp Speed” fast-track program announced that it would collaborate with seven businesses to produce COVID19 vaccines, including Johnson & Johnson, Moderna, Merck, Pfizer, and the University of Oxford in partnership with AstraZeneca [30].

From the above discussion, it is clear that most of the countries, international organizations, and charitable organizations engaged in the R&D of COVID vaccines are from the Western world. Currently, the TRIPS has been providing many IPs related to vaccines. TRIPS Article 7 explains the objectives in terms of protection and enforcement of the IPs as “the promotion of technological innovation,” “the transfer and dissemination of technology” to the mutual advantage of both “producers and users of technological knowledge,” and “social and economic welfare.” Article 8 obligates the member countries to protect public health and nutrition and promote the public interests congruent to the TRIPS Agreement provisions [31]. Moreover, it is the fundamental responsibility of sovereign governments to protect their citizens' health and safety. The Article 73 of the TRIPS Agreement may justifiably be invoked to override IP protections because the pandemic constitutes an emergency in international relations within the meaning of Article 73 (b) [32].

Brooke and Sherris [33] had argued that the availability of vaccines, particularly in the low and middle-income countries, depends mainly on the prior evaluation by the developed countries/regions like the US or European drug regulatory agencies. Moreover, the pharmaceutical manufacturers used to receive a large chunk of revenues from the developed countries. Therefore, there are scanty financial incentives available if the same is not sold in the same markets. Additionally, poorer countries' health agencies used to take green signals from the developed countries before approving/not approving the new products in the market. Though this is an independent regulatory approval guaranteeing the safety and effectiveness before the use, under such paradigms, the TRIPS can still become a hurdle for the availability of vaccine technology.

Guimon et al. [34] stated that the pandemic will not recede until the COVID-19 vaccine is viewed as a global public good. Even the UNAIDS Executive Director Winnie Byanyima, in an open letter to the global pharmaceutical industry leaders, also called on the global pharma industry “to unlock the secrets to their COVID-19 vaccine technologies” to produce a cheap and accessible “People's Vaccine” and not a profit vaccine [35]. Even a working paper by WTO staff highlighted that the evidence-based debate on the scope and effect of the TRIPS policy options is a task more important today than ever [36].

## 4. Discussion

### 4.1. Global Health Diplomacy: India's Role at the WTO Platform

The outbreak of COVID-19 had taken place in December 2019 in Wuhan, China. Consequently, the same was declared a Public Health Emergency of International Concern (PHEIC) and “Pandemic” by the WHO on January 30 and March 11 in 2020, respectively [37]. Concomitantly, the WTO has also cautioned that the “Pandemic represents an unprecedented disruption to the global economy and world trade, as production and consumption are scaled back across the globe.” The absence of vaccines/medicines for the ongoing pandemic became a more critical challenge for the entire globe. In this scenario, there was an overwhelming consensus for international collaboration to expedite vaccine development, manufacturing, a supply of effective medical technologies to ensure the protection of all patients across the globe. Even heads of several states urged the world leadership to treat the COVID-19 medical products as global public goods.

India has been known as the world's pharmacy, given its role in producing generic medicines [38]. Global health diplomacy has remained an important part of India's foreign policy. India has pursued the same at the peak of the pandemic. It had provided more than 150 countries with a wide range of medical and healthcare services, including medicines (hydroxychloroquine and paracetamol) and vaccines (Covishield and Covaxin). It has also collaborated with international organizations for vaccine R&D. It has contributed to the Global Alliance for Vaccines and Immunization (GAVI) [39].

In this backdrop, once again realizing the gravity of the situation, India and South Africa proposed a temporary waiver (IP/C/W/669) before the WTO's TRIPS Council as part of its global health diplomacy to expedite the development of medicines, vaccines, and diagnostics for prevention, containment, and treatment of COVID-19 [2]. Furthermore, the proposal casts a wide net, as practically any medical device required to diagnose, treat, or prevent COVID-19 could be eligible for such a waiver [40]. More than 350 civil society organizations and activists worldwide asked WTO member countries to support the Indian and South African joint proposal. Under the proposal's provisions, countries need to “waive off” the patents, copyrights, and other IPs not only for the products themselves but also for their underlying technologies—without facing WTO charges or penalties for violation of international trade rules. To take the lead further, India and South Africa had argued before the Council for TRIPS that “Given the current global emergency, WTO Members must work together to ensure that intellectual property rights such as patents, industrial designs, copyright, and the protection of undisclosed information do not obstruct timely access to affordable medical products such as vaccines and medicines, or the scaling-up of research, development, manufacturing, and distribution of medical products essential to combat COVID-19” [2]. Many access-to-medicines movements were organized by patient activists, civil society, and health-right groups who stood up to governments' passivity in the past to resist the pharmaceutical industry's monopolies for HIV medicines and eventually succeeded in gaining patent relief. These movements have resulted in a significant decrease in the prices of HIV medicines (over $10,000/person/year) dropped by 99% over a decade by allowing generic drugs in developing countries. Currently, the COVID-19 pandemic situation also presents a similar situation as the pandemic has affected every nation. Though in the case of HIV epidemic, it affected the global south more than the north and thus the support came in from the rich nations in Western Europe and North America. However, in the current COVID-19 pandemic, the rich nations have been affected more, with more cases and deaths resulting in global competition, lack of solidarity, and nationalist movements in addressing the domestic economic and health crises. There is a lack of global leadership and international cooperation in the current scenario, with geopolitical shifts leaving behind the interests of the developing nations. Hence, in this current scenario, vaccine nationalism has taken precedence over global cooperation and solidarity. Therefore, if the TRIPS waiver proposal is approved, the access to essential COVID-19 medicines, technologies, and diagnostics will improve drastically [41].

The proposal was also supported by UNAIDS, UNITAID, MSF (Medecins Sans Frontieres), academics, researchers, and numerous civil society organizations [42]. The WHO wholeheartedly lent its support to the Indian and South African proposal. WHO chief had welcomed India and South Africa's proposal and said “To ease international & intellectual property agreements on #COVID19 vaccines, treatments & tests to make the tools available to all who need them at an affordable cost.” The Indian leadership/health authorities realized that IPs are becoming barriers in the way of “scaling up production of test kit reagents, ventilator valves, N95 respirators, therapeutics, fluorescent proteins and other technologies used in the development of vaccines, etc.” Moreover, the waive-off argument has been advanced, realizing that the existing flexibilities in the TRIPS Agreement are “not adequate to address the fast-changing landscape of COVID19.” The fact that provisions under “compulsory licenses” are limited only to pharmaceutical products rather than the crucial medical devices required for combating the ongoing pandemic. The existing system became extremely onerous and time-consuming and of no practical use when exporters and importers have to comply with the existing provisions. In this backdrop, the joint proposal argued that the IP waiver has been very important, particularly for the developing countries with insufficient or no manufacturing capacities/finance for producing the vaccines/medicines [43]. However, these two are correlated but ultimately different problems. However, the financial resources are currently being raised for ensuring sufficient doses, but not the manufacturing capacities.

However, the proposal did not go through, given the rejection and lack of consensus among the developed countries. Rather, the WTO members have been divided into three groups. The first category including Chad, Tanzania, other African nations, Southeast Asia, and South American countries supported the proposal on behalf of the LDC countries and African Group. The second group of countries (China, Costa Rica, Chile, Columbia, Jamaica, El Salvador, Senegal, etc.) welcomed the proposal, but they did seek more clarifications. The third category comprises developed countries like Brazil, Canada, Norway, the UK, the US, Switzerland, and the EU, which outright rejected the proposal [42]. Chattu et al. have highlighted that though it is easy to talk of inequalities and inequities and include them in policies, and further added that, here is an opportunity for the world to show its solidarity for “Health For All” and nations should strive to find solutions to ensure equitable access to the COVID-19-related drugs, medical supplies, and vaccines [41].

From the above discussion, it becomes crystal clear that most vaccine R&D has been taking place in the developed countries' private and public institutions as it requires huge investments. However, at this juncture, the question is moot: which is more important, making money or saving a human life? This is weighing heavily on the minds of the public, especially in light of the ongoing critical issues of health and human security. Surprisingly, the developed countries, which are viewed as the main advocates of egalitarianism, democracy, health, and human rights by the global community, have not supported this humanitarian cause in the larger context. These 35 developed countries Australia, Brazil, Canada, Japan, Norway, Switzerland, the UK, the US, and the EU (27-member block) have rejected India's and South Africa's proposal. However, the other 100 nations have welcomed or fully supported it. This disagreement has resulted in rich vs. poor in the race of getting access to the COVID-19 medical equipment, treatment, and vaccines [43].

Have the TRIPS become a tool for the expansion of capitalism? Are these countries concerned about the 20 illnesses that can be prevented or treated, including COVID-19? If this is the case, why not put the question of returns, remuneration, profits, and so on to the side for the time being and focus on considerations, sensitivities, and humanitarian cause when whole humanity is suffering due to lack of access to COVID-19 vaccines and medicines?

To substantiate the above argument, it can be seen through the prism of deaths of millions of people due to infectious diseases every year. These diseases are perceived to be preventable or treatable. About 45% of deaths in Africa and Southeast Asia have occurred due to infectious diseases [44]. The death toll is unprecedentedly and unacceptably high in developing and the least countries. In the context of African nations, which depend on the development aid from rich nations, it would be prudent for the Africa Centers for Disease Control and regional bodies to embrace global health diplomacy to strengthen their capacity for disease preparedness and response [45]. During this crisis, the developing countries, especially in Asia and Africa, need to realign themselves and strengthen their health systems. A recent systematic review by Chattu et al. has emphasized that African Union needs to refocus and prioritize the continent's health challenges by innovatively adapting the canons of GHD towards attracting more funding and developing collaborative partnerships with relevant actors in the global health domain [46]. Although, the health crisis is due to given interlinked factors such as lack of healthcare facilities, poverty, unemployment, lack of sanitation but the critical factor for the same is unaffordability [47], inaccessibility, monopolization of production, and distribution of vaccines/medicines in the backdrop of the agreement on TRIPS.

On public health, trade, human rights, and the environment, governments seem to have lost faith in the value of working together. As highlighted by Jones Bruce, in the absence of credible great-power leadership from the US or China, the “middle powers” such as France and Germany have led to coordinating health and economic responses. Though the concept of “middle powers” is imprecise and inchoate, it refers to nations from the top 20 economies and lack large scale military power (or chose not to have a lead role) and is energetic in diplomatic and multilateral affairs such as France, Canada, Netherlands, Sweden, Germany, and the United Kingdom which were trying to fill the gaps in the international leadership [48]. They have shown their commitment and dedication by raising over $14 billion for providing free vaccines through the Vaccine Alliance to the countries that cannot afford them [49]. As Gostin et al. highlight the complexity of global health coordination and universal access to the COVID-19 vaccine, global health law's role is very critical as it supports global solidarity and reaches agreements to secure equitable access [50]. Moreover, there is an immediate need for cooperation and collaboration, an understanding of shared responsibility, and critical aspects such as transparency, accountability, trust, and fairness to overcome this COVID-19 pandemic [51].

## 5. Conclusions

COVID-19 had left indelible imprints and taught us several lessons such as the importance of global solidarity, international cooperation, and focusing on inequities and inequalities exposed during the ongoing pandemic. Given the monopoly of private ownership over vaccines/medicines/medical technology, the aspects of access and affordability to essential health care services will be compromised, violating the universal right to health. During this COVID-19 pandemic, the numerous facets of many healthcare systems' unpreparedness and fragile state were exposed. India, with its good infrastructure for pharmaceutical production and development, can become a hub for supplying generic medicines and essential medical equipment to the world, thereby improving access to the essential drugs, medicines, kits, and vaccines in many low- and middle-income countries (LMICs). There is a great need for cooperation and support from the developed nations to ensure the enjoyment of “right to health” by everyone. India must engage in global health diplomacy with a variety of global players to circumvent or obtain specific waivers for intellectual property rights (IP/IPRs) to safeguard the supply of life-saving and necessary pharmaceuticals and vaccines while maintaining equity and fairness. Every citizen has the right to health and human security. Therefore, the IP regime should not become a barrier to the availability and affordability of COVID-19 medical equipment and vaccinations. A large group of intellectuals, social activists, altruistic people, civil society organizations, nongovernmental organizations, international organizations, and other LMICs consider IPRs for COVID-19 essentials to be barriers during this pandemic. Hence, the countries that rejected the joint proposal of TRIPS waiver by India and South Africa should reconsider. Furthermore, those countries that claim to be strong supporters of human rights, egalitarianism, democracy, global health, and human security must rise to the occasion and lend their full support to India at the WTO for this great cause that prioritizes humanity over the business interests of the pharmaceutical industry.

## Data Availability

The data presented in this study are available on request from the corresponding author.
